# Effect of a neural relay on liver regeneration in mice: activation of serotonin release from the gastrointestinal tract

**DOI:** 10.1002/2211-5463.12382

**Published:** 2018-01-31

**Authors:** Ryosuke Inoue, Kenya Kamimura, Takuro Nagoya, Norihiro Sakai, Takeshi Yokoo, Ryo Goto, Kohei Ogawa, Yoko Shinagawa‐Kobayashi, Yukari Watanabe‐Mori, Akira Sakamaki, Satoshi Abe, Hiroteru Kamimura, Norio Miyamura, Hiroshi Nishina, Shuji Terai

**Affiliations:** ^1^ Division of Gastroenterology and Hepatology Graduate School of Medical and Dental Sciences Niigata University Japan; ^2^ Department of Developmental and Regenerative Biology Medical Research Institute Tokyo Medical and Dental University Japan

**Keywords:** gastrointestinal tract, hormone, liver regeneration, neural relay, serotonin

## Abstract

The development of therapeutic options to promote hepatic regeneration following severe liver injury is essential. While humoral factors have been reported as mechanisms of liver regeneration, the contributions of interorgan communication to liver regeneration have not been reported. In this study, we examined the effect of a neural relay on liver regeneration via activation of serotonin release from the gastrointestinal (GI) tract. Our results demonstrated that the afferent visceral nerve from the liver activates the efferent vagus nerve from the brain, leading to activation of serotonin release from the GI tract and contributing to liver regeneration. While it is difficult to apply these results directly to human health, we believe that this study may represent a step toward developing essential therapeutics to promote liver regeneration.

**Abbreviations**
BrdU: 5‐bromo‐2′‐deoxyuridine
Cap: capsaicin
GI: gastrointestinal
HGF: hepatocyte growth factor
HV: hepatic vagotomy
IL‐6: interleukin‐6
N.S.: not significant
PCNA: proliferating cell nuclear antigen
PH: partial hepatectomy
TPH1: tryptophan hydroxylase 1

The development of therapeutic options to promote hepatic regeneration following severe liver injury is important. It has been reported that in addition to humoral factors 1, 2, 3, 4, 5, 6, 7, 8, 9, 10, 11, 12, 13, 14, 15, the autonomic nervous system is also involved in hepatic regeneration 16, 17, 18. Many studies have examined the direct feedback between the brain and liver, starting from the liver via the afferent sympathetic nervous system to the brain, and then to the liver the hepatic branch of the efferent vagus nerve 16, 17. Kiba *et al*. reported that efferent vagus nerve in subdiaphragmatic vagus nerve, but not hepatic vagus nerve containing more than 90% of afferent nerve from the liver, is involved in and contributes to hepatic regeneration in a direct feedback system 16, 18. Interestingly, this phenomenon occurs following destruction of the ventromedial hypothalamus, which is the center of the sympathetic nervous system, and leads to activation of the vagus nerve 19, 20. These results suggest the importance of vagus nerve activity for hepatic regeneration 16.

On the other hand, Kiba *et al*. also showed proliferation of pancreatic beta cells, extrapancreatic secretory cells, and epithelial cells in the gastrointestinal (GI) tract was activated in vagus nerve‐activated mice 21, 22. These results suggest that vagus nerve activation after liver injury activates cell proliferation in multiple organs. Furthermore, it is suggested that various hormones produced in the GI tract cells are also activated via the vagus nerve. Lai *et al*. 23 showed that the combined administration of glucagon and insulin was effective for hepatic regeneration in rats that had undergone partial hepatectomy (PH). These results suggest that during liver damage, not only direct liver–brain feedback but also feedback between other organs activated by the vagus nerve may contribute to hepatic regeneration through the organ network from liver to brain and intestine, and to the liver via a neural relay. While the effector in this neural relay has not yet been determined, GI hormones are known to play an important role in hepatic regeneration.

In this study, we focused on serotonin released from chromaffin cells in the intestine, as this is known to be an important factor to encourage proliferation of liver cells 24, 25, 26, 27, 28. Interestingly, it was reported that mice deficient in tryptophan hydroxylase 1 (TPH1), an enzyme that synthesizes serotonin in chromaffin cells in the intestines, exhibit poor regeneration after hepatectomy 26. However, no reports have clarified the mechanisms by which serotonin secretion is activated and functions after liver injury through a neural relay.

Therefore, this study aimed to examine whether a neural relay plays a pivotal role in liver regeneration after liver injury, and whether serotonin contributes to liver regeneration after PH via this neural relay. Our study demonstrated that serotonin activation in the GI tract contributes to hepatic regeneration through a neural relay starting from liver to brain, to GI tract and to the liver.

## Materials and methods

### Animals

All animal experiments were approved by and conducted in full compliance with the regulations of the Institutional Animal Care and Use Committee at Niigata University, Niigata, Japan. Male C57BL/6JJcl mice (*n* = 120, 8 weeks of age, 25–30 g) purchased from CLEA Japan, Inc. (Meguro‐ku, Tokyo, Japan) were housed under standard conditions at temperature of 20–23 °C and humidity of 45–55%, in specific pathogen‐free facilities, and fed a standard diet.

### Development of animal models

The mice were divided into four groups (Fig. 1): control, sham‐operated mice; PH, in which PH was performed; Cap + PH, in which direct topical application of capsaicin was utilized to deafferentate the afferent visceral nerve; and HV + PH, in which transection of the hepatic branch of vagus nerve was performed. PH was performed by removing two‐thirds of normal liver tissue as previously described 29 at 10 weeks of age. Each of the five mice for each group was analyzed at the appropriate time points shown in Fig. 1. For PH, briefly, a midline skin incision was made on the mice under general anesthesia by intraperitoneal injection of pentobarbital sodium (Kyoritsu Seiyaku Corporation, Chiyoda‐ku, Tokyo, Japan) at a dosage of 40–50 mg·kg^−1^. For the selective afferent visceral nerve blockade, direct topical application of capsaicin (Wako Pure Chemical Industries, Osaka, Japan) dissolved in olive oil (50 mg·mL^−1^) was utilized to deafferentate the visceral nerve which contains afferent sympathetic fibers from the hepatobiliary system 30. This method was reported to show no effect on the other nerves, including vagus nerves 31. For selective afferent vagus nerve blockade, transection of the hepatic branch of vagus nerve, including more than 90% of afferent vagus nerve from the liver 16, 32, was performed.

**Figure 1:** Animal models and protocol. (A) Four groups of animal model were established: control group (Cnt), in which peritoneum incision was performed as a sham operation; partial hepatectomy group (PH), in which partial hepatectomy was performed; partial hepatectomy following visceral nerve block group (Cap + PH); and partial hepatectomy following vagus nerve block group (HV + PH). (B) For each group, tissues were collected, and expression of serotonin in the small intestine, BrdU uptake, PCNA expression in the liver, and liver weight‐to‐body weight ratio were assessed at appropriate time points. (C) Visceral nerve block was performed by applying capsaicin (Cap) to the sympathetic nervous plexus surrounding the celiac artery. Blockade was confirmed by immunostaining of the nerves with anti‐CGRP antibody.

### Histological analysis

Tissue samples for immunohistochemical staining were collected at appropriate time points after the procedures from each group and fixed in 10% formalin upon tissue collection before embedding in paraffin. A total of five different sections (10 μm) were cut from each of the five mice, and standard immunohistochemistry was performed using mouse anti‐insulin monoclonal antibody (I2018; Sigma, St. Louis, MO, USA), VECTASTAIN Elite ABC mouse IgG kit (PK‐6102; Vector Laboratories, Burlingame, CA, USA), and DAB chromogen tablets (Muto Pure Chemicals, Tokyo, Japan) for pancreatic beta cells.

Images were captured from each tissue section randomly, and number and size of the islet were measured by imagej software (version 1.6.0_20; National Institutes of Health, Bethesda, MD, USA).

For hepatocytes, anti‐PCNA antibody (2586; Cell Signaling Technology Japan, Tokyo, Japan), VECTASTAIN Elite ABC mouse IgG kit (PK‐6102; Vector Laboratories), and DAB chromogen tablets (Muto Pure Chemicals) were used. For small intestinal tissues, anti‐serotonin monoclonal antibody (M0758; DAKO, Santa Clara, CA, USA), VECTASTAIN Elite ABC mouse IgG kit (PK‐6102; Vector Laboratories), and DAB chromogen tablets (Muto Pure Chemicals) were used. For visceral nerves, anti‐CGRP monoclonal antibody (4901; Abcam, Cambridge, UK), VECTASTAIN Elite ABC rabbit IgG kit (PK‐6101; Vector Laboratories), and DAB chromogen tablets (Muto Pure Chemicals) were used. Images were captured from each tissue section randomly, and a quantitative analysis was performed using imagej software (version 1.6.0_20; National Institutes of Health) 33.

### BrdU *in situ* detection

Mice were injected intraperitoneally with 1 mg of BrdU (550891; BD Biosciences, Franklin Lakes, NJ, USA), 24 h before liver collection. Livers from five mice in each group were then collected and fixed in 10% formalin before embedding in paraffin. The labeled cells were immunostained with anti‐BrdU antibody, and BrdU In Situ Detection Kit (551321; BD Biosciences) was used for detection. BrdU‐positive cells in the liver were counted in each section, and images were captured from each tissue section randomly and a quantitative analysis was performed using imagej software (version 1.6.0_20; National Institutes of Health) 33.

### Serum cytokines

Blood samples were collected at appropriate time points, and serum was used to analyze the levels of IL‐6 and HGF by enzyme‐linked immunosorbent assay using a mouse IL‐6 ELISA Kit (KMC0061; Thermo Fisher Scientific, Waltham, MA, USA) and Quantikine HGF ELISA Kit (MHG00; R&D Systems, Minneapolis, MN, USA).

### Statistics

The data of histological analyses and liver body weight were statistically evaluated by two‐way factor repeated‐measures analysis of variance followed by Bonferroni's multiple comparison test by graphpad prism7 software (version 7.03; MDF, Tokyo, Japan).

## Results

### Development of animal models

Details of the animal groups are shown in Fig. 1. PH was performed as previously described 29. For selective afferent visceral nerve blockade, direct topical application of capsaicin (Cap) was utilized to deafferentate the afferent visceral nerve (Cap + PH) 30, and for selective afferent vagus nerve blockade, transection of the hepatic branch of vagus nerve [hepatic vagotomy (HV)], which includes more than 90% of afferent nerve from the liver, was performed 16, 32 (HV + PH).

### Activation of neural relay following partial hepatectomy

To confirm the activation of the neural relay after PH, the increase in beta cells in the pancreas and its inhibition in the Cap + PH group were examined. The number of islets was recorded and analyzed for each size category (small, < 10 000 μm^2^; medium, 10 000–30 000 μm^2^; large, > 30 000 μm^2^) 0, 1, and 3 days after PH in each type of mouse using imagej software (Fig. 2A).

**Figure 2:** Vagus nerve activation after partial hepatectomy. (A) Representative images from a section of pancreatic islet immunohistochemically stained with anti‐insulin antibody 3 days after partial hepatectomy. The number of pancreatic islets was classified with the area and was recorded for each size category (< 10 000 μm^2^, 10 000–30 000 μm^2^, and > 30 000 μm^2^) 0, 1, and 3 days after partial hepatectomy in the Cnt (B) and PH (C) groups. (D) Time‐dependent change of the number of small islets in the pancreas in the Cnt, PH, Cap + PH, and HV + PH groups. Five different pancreatic sections from each of the five mice in all groups were immunohistochemically stained with anti‐insulin antibody, and a quantitative analysis was performed using imagej software. The values represent mean ± SD (*n* = 25 for each group). *P < 0.05, ***P < 0.001, and N.S., no statistical significance compared with the Cnt group. Two‐way factor repeated‐measures analysis of variance followed by Bonferroni's multiple comparison test.

Three days after PH, modifications to islet size showed a significant increase in the proportion of small‐sized islets (1 day after: 58.0 ± 3.0% vs 67.0 ± 2.4%, *P* < 0.05; 3 days after: 58.1 ± 4.4% vs 71.7 ± 3.6%, *P* < 0.001), while medium‐sized islets showed a mild decrease (1 day after, 27.0 ± 3.7% vs 19.6 ± 1.4%, N.S.; 3 days after, 27.6 ± 2.8% vs 15.7 ± 2.5%, N.S.), although this was not significant. Large‐sized islets showed no significant difference between the two groups (1 day after, 14.9 ± 1.2% vs 13.3 ± 3.1%, N.S.; 3 days after, 13.4 ± 2.6% vs 12.3 ± 1.1%, N.S.) (Fig. 2B,C). Time‐dependent changes of small‐sized islets in the control, PH, Cap + PH, and HV + PH groups showed a significant increase in the PH group and inhibition by visceral nerve blockade in the Cap + PH group, with relatively weaker inhibition in the HV + PH group (Fig. 2D).

These results provide evidence that the efferent vagus nerve was activated after PH and that the afferent visceral nerve is important to send a signal to the central nervous system.

### Effect of neural relay on DNA synthesis in hepatocytes after partial hepatectomy

To examine the effects of the neural relay on liver regeneration, DNA synthesis in hepatocytes was analyzed by immunostaining with anti‐BrdU antibody (Fig. 3A,B). Quantitative analysis showed that 37.3 ± 4.7% and 22.3 ± 2.5% of hepatocytes were positively stained for BrdU in a high‐power field 2 and 3 days after PH, respectively, which were significantly higher than that of the control group (2.7 ± 0.6%, *P* < 0.001, 1.3 ± 0.6%, *P* < 0.001). To examine the role of the afferent neural relay, the same set of analyses were performed in the Cap + PH and HV + PH groups. A significant inhibition in the increase in BrdU‐positive cells was observed in the Cap + PH group 2 and 3 days after the procedure (9.3 ± 2.1% and 6.7 ± 1.5%, respectively, both N.S. compared with the control group), while a similar level of increase in BrdU‐positive cells was seen in the HV + PH group compared with the PH group 2 and 3 days after the procedure (31.7 ± 3.5% and 21.0 ± 2.0%, respectively, both *P* < 0.001 compared with the control group) (Fig. 3B). No differences were seen between the groups later than 5 days after the procedure. These results suggest that the neural relay is significantly related to DNA synthesis after PH and that the afferent visceral nerve contributes to relay the signal. The hepatic vagus nerve showed a lower effect on DNA synthesis in hepatocytes.

**Figure 3:** Effect of neural relay on DNA synthesis in hepatocytes after partial hepatectomy. (A) Representative images of BrdU‐positive cells in the liver. (B) Time‐dependent change of the number of cells positively stained for BrdU in the Cnt, PH, Cap + PH, and HV + PH groups. Five different sections from each of the five mice in all groups were immunohistochemically stained with anti‐BrdU antibody, and a quantitative analysis was performed using imagej software. The values represent mean ± SD (*n* = 25 for each group). ***P < 0.001, and N.S., no statistical significance compared with the Cnt group. Two‐way factor repeated‐measures analysis of variance followed by Bonferroni's multiple comparison test.

### Effect of neural relay on hepatocyte proliferation after partial hepatectomy

To examine whether the neural relay contributes to hepatocyte proliferation after PH, the number of proliferating cell nuclear antigen (PCNA)‐positive cells was assessed by staining. Quantitative analysis showed that 14.3 ± 3.1%, 44.3 ± 7.6%, and 38.3 ± 3.8% of hepatocytes were positively stained for PCNA in a high‐power field 1, 2, and 3 days after PH, respectively (Fig. 4A,B), which were significantly higher than that of the control group (6.3 ± 1.5%, *P* < 0.001; 5.0 ± 3.5%, *P* < 0.001; and 7.3 ± 1.5%, *P* < 0.001, respectively). To examine the role of the afferent neural relay, the same set of analyses were performed in the Cap + PH and HV + PH groups. A significant inhibition in the increase in PCNA‐positive cells after PH was observed in the Cap+PH group 2 and 3 days after the procedure (25.3 ± 3.2% and 25.7 ± 6.8%, respectively), although this was higher than that of the control group. The HV+PH group showed a similar level of activation of hepatocyte proliferation compared with the control group 2 and 3 days after the procedure (42.7 ± 5.7%, *P* < 0.01, and 36.7 ± 3.1%, *P* < 0.01 compared with the control group, respectively) (Fig. 4B). No significant differences between the groups were seen later than 5 days after the procedure. These results suggest that the neural relay is significantly related to hepatocyte proliferation after PH and that the afferent visceral nerve contributes to relay the signal. The hepatic vagus nerve showed a lower effect.

**Figure 4:** Effect of neural relay on hepatocyte proliferation after partial hepatectomy. (A) Representative images of PCNA‐positive cells in the liver. (B) Time‐dependent change of the number of cells positively stained for PCNA in the Cnt, PH, Cap + PH, and HV + PH groups. Five different sections from each of the five mice in all groups were immunohistochemically stained with anti‐PCNA antibody, and a quantitative analysis was performed using imagej software. [Correction added after online publication on 14 February 2018: anti‐BrdU antibody changed to anti‐PCNA antibody]. The values represent mean ± SD (*n* = 25 for each group). *P < 0.05, **P < 0.01, ***P < 0.001, and N.S., no statistical significance compared with the Cnt group. Two‐way factor repeated‐measures analysis of variance followed by Bonferroni's multiple comparison test.

### Effect of neural relay on liver volume recovery after partial hepatectomy

To examine the effect of the neural relay on the recovery of liver volume, time‐dependent liver weight after PH was assessed. As expected, the PH group showed recovery of liver weight‐to‐body weight ratio 3 days (4.2 ± 0.2%) and 5 days (4.8 ± 0.4%) after PH to the same level as that of the control group (N.S.). The HV + PH group showed similar results 3 days (4.7 ± 0.1%) and 5 days (4.7 ± 0.03%) after PH, while the Cap + PH group showed a significant delay in recovery 3 days (3.1 ± 0.2%, *P* < 0.001) and 5 days (3.8 ± 0.1%, *P* < 0.001) after PH (Fig. 5). The Cap + PH group showed a relatively slower recovery even after 5 days, and humoral growth factors such as hepatocyte growth factor (HGF) remained significantly higher in this group compared with the other three groups 7 days after the procedure (Fig. S1).

**Figure 5:** Effect of neural relay on liver weight‐to‐body weight ratio after partial hepatectomy. Time‐dependent changes of liver weight‐to‐body weight ratio after partial hepatectomy in the Cnt, PH, Cap + PH, and HV + PH groups. Liver weight (LW)‐to‐body weight (BW) ratio was measured in each of the five mice from the four groups at appropriate time points. The values represent mean ± SD (*n* = 5 for each value). **P < 0.01, ***P < 0.001, and N.S., no statistical significance compared with the PH group. Two‐way factor repeated‐measures analysis of variance followed by Bonferroni's multiple comparison test.

These results suggest that the neural relay is significantly associated with recovery of liver volume after PH via the afferent visceral nerve and not via the hepatic vagus nerve plexus.

### Activation of serotonin release from intestinal cells following partial hepatectomy

To determine the factors contributing to liver regeneration after PH in this neural relay, various GI hormones activated by the efferent vagus nerve were tested. Activation of serotonin expression in the enterochromaffin cells in the small intestine was monitored in a time‐dependent manner after PH in the groups.

Immunohistochemical staining was performed using an anti‐serotonin antibody, and the amount of serotonin in the enterochromaffin cells was assessed (Fig. 6A,B). Quantitative analysis showed 6.1 ± 0.3%, 6.1 ± 0.2%, and 5.6 ± 0.2% of small intestinal mucosal epithelium cells stained positively for serotonin 1, 2, and 3 days after PH, which were statistically higher than that of the control group (3.9 ± 0.6%, *P* < 0.001; 4.2 ± 0.3%, *P* < 0.001; 4.2 ± 0.5%, *P* < 0.01) (Fig. 6B). These results suggest that serotonin was induced by PH.

**Figure 6:** Activation of the serotonin release from the enterochromaffin cells after partial hepatectomy. (A) Representative images of serotonin‐secreting enterochromaffin cells in the small intestine of each group. Expression of the serotonin was confirmed by immunostaining of the cells with anti‐serotonin antibody. (B) Time‐dependent change of the number of cells positively stained for serotonin in the Cnt, PH, Cap + PH, and HV + PH groups. Five different sections from each of the five mice in all groups were immunohistochemically stained with anti‐serotonin antibody, and a quantitative analysis was performed using imagej software. [Correction added after online publication on 14 February 2018: anti‐insulin antibody changed to anti‐serotonin antibody]. The values represent mean ± SD (*n* = 25 for each group). **P < 0.01, ***P < 0.001, and N.S., no statistical significance compared with the Cnt group. Two‐way factor repeated‐measures analysis of variance followed by Bonferroni's multiple comparison test.

To examine the role of the afferent neural relay, the same analyses were performed in the Cap + PH and HV + PH groups. In the visceral nerve block group (Cap + PH), an increase in serotonin level in the small intestine was not seen compared with the control group (1 day after, 4.7 ± 0.3%; 2 days after, 4.8 ± 0.3%; 3 days after, 4.6 ± 0.3%), indicating suppression of serotonin in the enterochromaffin cells after PH when the afferent visceral nerve was blocked. In addition, vagus nerve block (HV + PH) showed an increase in serotonin levels to the same level as the PH group (1 day after, 5.3 ± 0.6%; 2 days after, 5.5 ± 0.1%; 3 days after, 5.5 ± 0.5%), indicating no significant association of the afferent vagus nerve in the neural relay from the liver toward the central nervous system to stimulate serotonin (Fig. 6B). These results suggest that PH induced activation of the neural relay through afferent visceral nerves through to the efferent vagus nerve which contributes to increased serotonin expression in the enterochromaffin cells. This leads to an increase in DNA synthesis in the hepatocytes, hepatocyte proliferation, and recovery of liver volume.

## Discussion

Development of therapeutic options to promote hepatic regeneration following severe liver injury is needed. To date, many studies on the mechanisms of hepatic regeneration have investigated various growth factors 5, 6, 7, 8, 9, 10, 11, 12, 13, 14, cytokines 1, 2, 3, 4, 15, signal transducers 34, 35, GI hormones 23, 24, 25, 26, 27, 28, and direct feedback of autonomic nerves 16, 17, 18, which are considered to play an important mechanistic role in homeostasis in various organs. These nerves are distributed in various internal organs including blood vessels, heart, lungs, GI tract, liver, and reproductive organs and are controlled by a feedback system situated predominantly in the brain, playing important organ‐related roles as a network for maintaining homeostasis 36.

The importance of the efferent vagus nerve in hepatic regeneration was reported by Kiba *et al*. They created a mouse model of vagus nerve activation by destroying the center of the sympathetic nervous system with no direct liver damage 19 and showed the same level of hepatocyte proliferation to that seen after PH 16, 17, 18. In addition, vagus nerve activation following PH increased pancreatic beta cells 37, 38, 39. We also confirmed the same effect in our study by activating the vagus nerve using sympathetic nerve destruction 21, 31, 40 (Fig. 1). These results suggest that the neural signal relay from the liver to the efferent vagus nerve is important for hepatocyte proliferation and maintenance of blood glucose level following liver injury. However, no study has focused on the network of these organs through the neural relay, the afferent signal from the injured liver, or the effector for liver regeneration in this neural relay.

On the other hand, interorgan communication functions in a coordinated manner as a biological mechanism to maintain homeostasis in living organisms and is very important in various pathologies. For example, studies into the relationship between the GI tract and the brain have shown intestinal bacterial flora to be strongly involved in Parkinson's disease 41 and autism 42.

Therefore, our study aimed to investigate whether a neural relay contributes to liver regeneration depending on communication with other organs, such as the GI tract. To confirm the contribution of a neural relay, we utilized a neural blockade procedure (Fig. 1), and to examine the association of the GI tract, efferent vagus nerve activation was confirmed upon liver injury (Fig. 2) followed by analysis of serotonin levels and liver regeneration. Serotonin is a monoamine neurotransmitter that is mostly found in chromaffin cells in the intestine 24, 25. Release of serotonin from the GI tract increases when the parasympathetic nervous system is activated 25. Serotonin is contained in platelet granules and is released when platelets come into contact with liver cells. It mediates 5‐HT_2_ receptors in the liver to function as a growth factor for liver cells 26, 27, 28. Lesurtel *et al*. analyzed mice lacking TPH1, which is the rate‐limiting enzyme for the synthesis of peripheral serotonin, and reported that platelet‐derived serotonin mediates liver regeneration after hepatectomy. In addition, they found that failure to regenerate was rescued by reloading serotonin‐free platelets with a serotonin precursor molecule 26. Similar results have been reported by others: Murata *et al*. and Papadimas *et al*. found that the effects of serotonin on DNA synthesis were arrested by 5‐HT_2_ receptor blockade at the G_1_/S transition 13, 43; Balasubramanian *et al*. 44 reported induction of DNA synthesis in primary cultures of rat hepatocyte by serotonin; and Nocito *et al*. 27 used a normothermic hepatic ischemia model mouse. Matondo *et al*. 45 reported that a small amount of serotonin in the liver is sufficient for liver regeneration although the biological homeostasis was disturbed by serotonin transporter depletion. In addition, serotonin protected mouse liver from cholestatic injury by stabilizing the bile salt pool after bile duct ligation through adaptation of renal transporters in cholestasis 46. Reduced serotonin reuptake transporter function caused insulin resistance and hepatic steatosis independent of food intake 47. These reports support that serotonin functions to activate the proliferation and growth of the hepatocyte *in vitro* and *in vivo*. However, there have been no reports showing how serotonin release is activated after liver injury.

Our results demonstrated that the afferent visceral nerve, not the afferent vagus nerve, significantly contributes to the activation of the efferent vagus nerve upon liver injury and that the GI tract activates the release of serotonin by this signal relay and contributes to liver regeneration evidenced by BrdU (Fig. 3), PCNA (Fig. 4), and liver weight‐to‐body weight ratio (Fig. 5). A summary of our studies and the reported effect of autonomic nervous system are shown in Fig. 7. Other factors such as serum HGF (Fig. S1) and IL‐6 (Fig. S2) are also involved in liver regeneration and, interestingly, HGF remained at high levels after PH when the visceral nerve was blocked (Fig. S1). This result indicates that the afferent visceral nerve contributes to activation of hepatocyte proliferation through signaling, including serotonin, and HGF compensates for the delay in recovery of cellular growth (Figs 6 and S1).

**Figure 7:** Mechanism of hepatic regeneration through neural signal. (A) The direct feedback between the liver and the brain. (B) The involvement of GI tract in liver regeneration via the neural relay.

Further analyses are necessary to fully elucidate the mechanisms of liver regeneration after liver injury. However, our study demonstrates that the autonomic nervous system plays a pivotal role for liver regeneration to maintain homeostasis and interorgan communication between the liver and the GI tract upon liver injury (Fig. 7).

In conclusion, we report that a liver damage‐mediated neural relay causes the release of serotonin by the GI tract and this directly promotes hepatic regeneration. While it is difficult to directly apply these results to the human health, we believe that this study represents a step toward developing essential therapeutics to promote liver regeneration.

## Author contributions

RI, TN, NS, TY, RG, KO, and YSK performed experiments; KK, YWM, AS, SA, HK, and NM analyzed the data; KK, HN, and ST conceived and supervised the study; and KK and ST wrote the manuscript.

## Supporting information


**Fig. S1.** Time‐dependent changes of serum HGF after partial hepatectomy in the Cnt, PH, Cap + PH, and HV + PH groups.

**Fig. S2.** Time‐dependent changes of serum IL‐6 after partial hepatectomy in the Cnt, PH, Cap + PH, and HV + PH groups.
